# Advances in the Application of Liquid Chromatography in the Detection of Pollutants

This article has been retracted.

**DOI:** 10.1155/2022/2152615

**Published:** 2022-08-26

**Authors:** XinYu Hu

**Affiliations:** School of Food Science and Engineering, Shandong Agricultural University, Taian 271000, China

## Abstract

Food is easy to be contaminated because of its complex composition. Therefore, in order to protect people from potential food contaminants, it is very necessary to test for various contaminants in food. Liquid chromatography is widely used in the field of food safety detection. In addition, with the development of liquid chromatography technology, more and more new instruments are combined with liquid chromatography. Compared with traditional liquid chromatography, combined liquid chromatography has great advantages in efficiency and operation. Therefore, it is rapidly promoted in the field of food safety testing. In this paper, the results of the determination of three kinds of food pollutants by different liquid chromatography methods are reviewed, and the indexes are compared and analyzed.

## 1. Introduction

Food is a variety of finished products and raw materials for human consumption or drinking. It is a very complex compound composed of natural compounds (lipids, carbohydrates, proteins, minerals, vitamins, and trace elements). It is very important to ensure the safety of food. Food should be nontoxic and harmless, meet nutritional requirements, and not cause any acute, subacute, or chronic harm to human health. According to the definition of food safety by Benoy, food safety is “a public health problem of the effects of toxic and harmful substances in food on human health.”

Several of these compounds, such as contaminants from food processing, pesticide and veterinary drug residues, and contaminants from natural sources (mycotoxins, etc.), may also be harmful to human health, although they are usually present in small amounts. Countries around the world have formulated corresponding laws, regulations, and standards for various substances that appear in food.

In order to protect people from potential food hazards, detection and risk assessment of toxic and hazardous substances in food are required. It begins by obtaining data from reliable, fit-for-purpose analytical methods to estimate consumer exposure and ingestion levels of contaminants and residues [1]. Liquid chromatography (LC) is the most commonly used chromatographic method in the analysis of food. In addition, high sensitivity or high resolution can be obtained in combination with other novel detection devices such as mass spectrometry (MS) [2].

The purpose of this review is to describe the differences between different liquid chromatography methods for the determination of contaminants in food samples. It includes references to recently published papers on chromatography in the field of food safety, as well as the application of new technologies. We have listed three common food contaminants. Then, the differences in the determination methods and effects of different liquid chromatography techniques were discussed, and by comparing the chromatographic columns and other related factors, some suggestions were provided for the selection of liquid chromatography for the determination of food contaminants, in order to improve the separation effect of liquid chromatography.

## 2. Common Liquid Chromatography

Liquid chromatography technology has been widely used in food safety detection. Traditional liquid chromatography mainly includes paper chromatography and thin chromatography. With the development of chromatography technology, the combination of modern liquid chromatography and mass spectrometry has become the main trend today, with the advantages of high efficiency, rapidity, and convenience. In the field of food safety testing, modern liquid chromatography-mass spectrometry is regarded as a reliable quantitative analysis tool [3].

### 2.1. Traditional Liquid Chromatography

Traditional liquid chromatography mainly includes paper chromatography and thin chromatography.

The principle of paper chromatography is the principle of similar compatibility, which is analyzed by the dispersing speed of the split system in the same medium. Paper chromatography is less used in food safety testing because of its slightly inferior efficiency and separation effect. Paper chromatography is less used in food safety testing because of its slightly inferior efficiency and separation effect. Even if it is used, it is improved. For example, Fereshte Mohamadi et al. [4] established a three-dimensional paper chromatography (3D-PC) method for the determination of tartrazine and indigo carmine in food samples (colorimetric method).

Thin-layer chromatography is an analytical method in which an adsorbent and a support agent are uniformly coated on a glass or plastic plate to form a thin layer for chromatographic separation. Compared with paper chromatography, a wider range of corrosive color reagents, mobile phases, and stationary phases can be used than paper chromatography. Therefore, the application in the field of food safety detection is more extensive, and it can also be combined with mass spectrometry and fluorescence detection technology. For example, Claudia et al. [5] established a high performance thin-layer chromatography-fluorescence detection method to determine the emulsifier in food.

### 2.2. Liquid Chromatography-Mass Spectrometry

In the field of food safety testing, the most commonly used methods are liquid chromatography-mass spectrometry (LC-MS) and LC-MS/MS, which can realize the analysis of small molecular substances (approx <1200 Da), use traditional mass spectrometers (QqQ and TOF), or use a HRMS hybrid detector (QTOF or Q-Orbitrap, etc.). Sample clean-up techniques also play an important role in LC-MS methods, such as solid phase extraction (SPE) and immunoaffinity columns (IAC) and QuEChERs; in addition to electrospray ionization (ESI), atmospheric pressure chemical ionization (APCI) is also the most commonly used ionization mode for LC-MS methods [6].

In the detection of some types of substances, people often use high performance liquid chromatography-mass spectrometry (HPLC) to determine substances. HPLC is a more efficient separation chromatographic technique than ordinary LC, with high selectivity, sensitivity, and resolution [7]. The working principle of HPLC is shown in Figure 1.

HPLC is a chromatography analytical technique for the separation, quantification, and identification of a variety of compounds. Sample components can be effectively separated by pressurized liquid and sample mixture through a column filled with adsorbent. The principle is that components are separated from the stationary phase at different times based on hydrophilic or molecular mass, hydrophobic properties, or electric charge through the interaction of the column components with the appropriate type of stationary phase [8]. High performance liquid chromatography has also proved useful in the determination of contaminants in food [9]. Therefore, HPLC is widely used for quantitative analysis of a large number of compounds, including contaminants in food processing, pesticide and veterinary drug residues, and mycotoxins, to evaluate food quality. HPLC can also be used in combination with mass spectrometry (HPLC-MS or HPLC-MS/MS), fluorescence (HPLC-FD), or ultraviolet (HPLC-UV) detection techniques [10]. These methods have been widely used in the field of food safety testing.

## 3. Application of Liquid Chromatography in Determination of Food Contaminants

There are many kinds of foods, and their characteristics and nutritional components are more complex. Food may be contaminated by various chemical substances during production, transportation, and storage. Excessive amounts of some substances may endanger human health. Therefore, contaminant residues in food are also the focus of people's attention in recent years. With the wider application of HPLC in food safety testing, people can obtain information on various foods through it, which is helpful for people's healthy life.

Acrylamide, veterinary drugs, and mycotoxins are common contaminants in food. Moreover, these three kinds of food pollutants do great harm to the human body. Therefore, this paper analyzes and compares the test accuracy of different liquid chromatography methods based on the detection process and test results of these three common food contaminants. The chromatographic conditions of different chromatographic methods are summarized in Tables 1–3.

### 3.1. Analysis of Acrylamide

Acrylamide (AM) is formed during the thermal processing (i.e., frying and baking) of carbohydrate-rich foods and is one of the products of the Maillard reaction in the reaction of asparagine and sugars (glucose and fructose) [11]. The International Agency for Research on Cancer (IARC, 1994) has classified acrylamide (2-acrylamide) as a probable human carcinogen and has called it a neurotoxin for the World Health Organization (WHO, 2002). To this day, the content of acrylamide in foods has been of concern, especially in fried and baked goods containing carbohydrates and amino acids (asparagine) [12]. Therefore, it is necessary to use new liquid chromatography methods to determine the content of acrylamide in food. For the determination of acrylamide in food, the following section lists some different liquid chromatography methods.

#### 3.1.1. LC-MS/MS

Roach et al. [13] used an Extrasyl ODS1 (200 × 30 mm, 5 *μ*m) chromatographic column for the determination of acrylamide in potato chips by a reversed-phase LC-MS/MS method. It can be known from the original literature that the mobile phase they used is acetic acid-methanol-Milli-Q water (0.1 : 1.0 : 98.9), and the flow rate is 0.2 mL min^−1^. Cheong Tae et al. [14] improved the LC-MS/MS method and used it to determine the content of acrylamide in processed food. The selected chromatographic column is Aqua C18 HPLC (2 × 250 mm, 5 *μ*m particles). It is 0.2% acetic acid aqueous solution and 1% methanol, and the flow rate is 0.2 mL/min.

Eleonora et al. [15] used RP C18 column (Phenomenex, Torrance, CA, USA) in the QuEChERS extraction and LC-MS combined detection method established in the experiment of detecting the content of acrylamide in dried fruit (250 mm × 2 mm 5 *μ*m particle size) and edible seeds (Phenomenex, Torrance, CA, USA). They chose a pore size of 110 A based on the molecular weight of acrylamide (Mr = 71.078). The mobile phases chosen were 0.1% formic acid in water (99.5%, solvent A) and 0.1% formic acid in methanol (0.5%, solvent B) with a flow rate of 0.25 mL/min at ambient temperature.

#### 3.1.2. HPLC-MS/MS and HPLC-UV

Lubomir et al. [16] used HPLC-MS/MS for the determination of AM in thermally processed seafood using a shorter narrow-bore column (Phenomenex Synergi Fusion-RP C18 column 50 mm × 2 mm, 2.5 *μ*m), replacing traditional columns like those listed above (250 or 150 mm × 2 or 4.6 mm). Its polar endcaps operate in 100% water and provide acceptable retention and peak shape for acrylamide. In addition, the 50 mm column length reduces analysis time (only 8 minutes of run time, including wash and equilibration time per analysis). Mobile phase A consists of 5% methanol, 0.1% formic acid, and 95% water. Mobile phase B is methanol at a flow rate of 0.2 mL/min.

Haiyan et al. [17] used Hypersil ODS-C18 (250 mm × 4.6 mm, 5 *μ*m) (Thermo Scientific, Waltham, MA, USA) solvent A for the determination of acrylamide in Chinese baked or fried foods. With a mixture of 10% acetonitrile and 90% water containing 0.10% formic acid, solvent B was pure acetonitrile, and the flow rate was 0.40 mL/min.

### 3.2. Analysis of Veterinary Drugs

Veterinary drug residues are the residues formed in animal visceral tissues and their products (egg, milk, etc.) after veterinary drugs act on animals, which usually includes sulfonamides, antibiotics, and pesticides. Veterinary drug residues are one of the research hotspots in recent years, and all countries in the world have strengthened the detection of veterinary drug residues in international trade animal food. In this paper, representative sulfonamides will be selected as the research objects, and the effects and differences of different chromatographic methods will be discussed. For the determination of sulfonamides in food, the following section lists some of the different liquid chromatography methods.

#### 3.2.1. LC-MS/MS

The column used by Marisol et al. [18] in their LC-MS-MS analysis for the presence of sulfonamides in honey products was a Zorbax Eclipse XDB-98 (50 × 4.6 mm, 1.8 *μ*m), supplied by Agilent. Chromatographic separation was performed with 0.5% aqueous formic acid (mobile phase A) and ACN (mobile phase B) as mobile phases at a flow rate of 0.4 mL/min.

Petrarca et al. [19] used a Poroshell 120 HILIC column (150 × 3 mm, 2.7 *μ*m) in their LC-QTOF-MS analysis of sulfonamide antibiotic residues in meat and/or egg baby food (Agilent Technologies, Santa Clara, CA, USA). The mobile phase was 20 mM ammonium formate in water, pH 3 : methanol, 1 : 1 *v*/*v* (solvent A) and acetonitrile (solvent B) at a flow rate of 0.2 mL/min.

#### 3.2.2. HPLC and HPLC-MS/MS

Tian and Kaifeng [20] used Amethyst C18-H (250 × 4.6 mm, 5 *μ*m) as a chromatographic column in the simultaneous determination of sulfonamides in milk by in situ magnetic ionic liquid dispersion liquid-liquid microextraction-high performance liquid chromatography. A 0.5% sodium dihydrogen phosphate aqueous solution-acetonitrile (85 : 15, *v*/*v*) was used as the mobile phase, the flow rate was 2.0 mL/min, and the measurement wavelength of the UV detector was set to 270 nm for simultaneous detection.

Tao et al. [21] used an F5 column (50 × 3.0 mm, 2.6 *μ*m, Phenomenex, Torrance, CA, USA) for the detection of sulfonamide antibiotic residues in aquaculture by online solid-phase extraction-UHPLC-MS/MS. For chromatographic separation, the mobile phases of UHPLC were 0.1% formic acid water (A) and 0.1% formic acid ACN (B), and the total flow rate of the liquid phase was controlled at 0.45 mL/min.

Hoff et al. [22] used a high performance liquid chromatography column purrospher STAR C18 (150 × 4.6 mm, 5 *μ*m) for the determination of sulfonamide antibiotics and metabolites in animal liver, muscle, and kidney samples by HPLC-Qqlitm-MS/MS method. The mobile phase consisted of HPLC-grade water acidified with 10 mM formic acid and ACN acidified with 10 mM formic acid at a flow rate of 0.2 mL/min.

### 3.3. Analysis of Mycotoxins

Among the mycotoxins, aflatoxins are more typical. Aflatoxins (AFs) grow in food, including AFB1, AFB, AFG, and AFG2. They are toxic chemicals produced by a variety of fungi, which can cause a variety of food contamination and pose a threat to human health [23]. Likewise, the following section lists several different liquid chromatography methods for the detection of aflatoxins in foods.

#### 3.3.1. Analysis of LC-MS/MS

Purospher Star RP-18 column (50 × 2.1 mm, 2 *μ*m) was selected for the study by Abdallah et al. [24] for the detection of aflatoxin B in maize by LC-MS/MS. The mobile phase was 0.1% acetic acid-methanol (60 : 40) at a flow rate of 0.25 mL/min.

Ala' Yahya et al. [25] used a ZORBAX Eclipse XBD-C18 (100 × 2.1 mm, 1.8 *μ*m) for the determination of aflatoxins in food by the LC-ESI-QTOF-MS/MS method (PN. 928700-902) column at a flow rate of 0.3 mL/min. The mobile phase was 1% formic acid and 2 mM ammonium formate in water (A) and 1% formic acid in methanol (B).

#### 3.3.2. Analysis of HPLC-MS/MS and HPLC-FD/FLD

Riwei et al. [26] used Zorbax SB-C18 column (50 × 2.1 mm, 3.5 *μ*m) in the determination of aflatoxin in Ural licorice by HPLC-MS/MS, mobile phase A was water, eluent B is acetonitrile, both contain 0.1% formic acid, and the flow rate is 2 mL/min.

Nor Shifa and Bahruddin [27] used a C18 Hypersil gold (250 × 4.6 mm, 5 *μ*m) column for the determination of aflatoxins in milk by in-syringe dispersive microsolid phase extraction by HPLC-FD with the mobile phase of acetonitrile : methanol 3 : 2 (*v*/*v*) flow rate of 1.2 mL/min.

Fatma et al. [28] used ACE 5 C18, 100 A (250 × 4.6 mm, 5 *μ*m) in the determination of aflatoxins in pistachios and peanuts by HPLC-FLD, and the mobile phase was water-acetonitrile-ethanol (6/2/3, *v*/*v*/*v*); the flow rate is 2-3 mL/min.

## 4. Discussion

### 4.1. Analysis of Chromatogram Peaks

The flow rate is the main factor that affects the peak area of the final result chromatogram. Among all liquid chromatography methods for the determination of acrylamide, there are three methods (LC-MS/MS, improved LC-MS/MS, and HPLC-MS/MS) at similar flow rates. Under the condition that this factor remains unchanged, comparative analysis is carried out by comparing the final chromatograms. There are multiple chromatograms according to (and other peak resolution, peak symmetry, and sharpness) filter. The three methods all use the multiple reaction detection mode (MRM). Under different voltages, the transition changes of the ion collision energy are different, and the chromatograms under such conditions are also different. A comparison of the best chromatograms screened for each method is shown in Figure 2. By comparison, we found that the improved LC-MS/MS method has more symmetry in the shape of the chromatographic peaks than the LC-MS/MS method. It is much better and easier to calculate the peak area, and the HPLC-MS/MS method can produce peaks within two minutes and has good symmetry, so the HPLC-MS/MS method is an extremely useful method for the determination of acrylamide in food. The optimal method shortens the analysis time and improves the quality of sample analysis.

The best chromatographic peaks (Figure 3) for the determination of acrylamide content by HPLC-UV were produced when the mobile phase was 10% (*v*/*v*) acetonitrile at a flow rate of 0.40 mL/min. In both cases, 15% (*v*/*v*) acetonitrile with a flow rate of 0.40 mL/min and 10% (*v*/*v*) acetonitrile with a flow rate of 0.50 mL/min were not as effective as the first mobile phase and flow rate The chromatographic peaks produced by the selection are effective, so simply increasing the flow rate and the acetonitrile concentration cannot improve the chromatographic peaks.

In the experiment of determination of sulfonamides by liquid chromatography, the differences of the corresponding methods of different chromatographic peaks were analyzed under the condition that the flow rate was almost constant. In the experiment of the HPLC-QqLIT-MS/MS method for the determination of sulfonamides, there are 16 kinds of tested substances. In this experiment, two extraction methods, PLE and USE, were set up for comparison and verification. By observing the shape of their chromatographic peaks (Figure 4), Figure 4(a) is the chromatogram of the PLE method, and Figure 4(b) is the chromatogram of the USE method. From the symmetry, the degree of separation, and the sharpness of the different substances in the chromatogram, it is inferred that the chromatogram of the USE method is more accurate and precise. By comparing the shape of the chromatogram peaks, it is concluded that the USE method is more accurate than the PLE method, and this conclusion has also been confirmed by Valente et al. in the laboratory for many years.

In the determination of sulfonamides in food by the HPLC-QqLIT-MS/MS method and in situ magnetic ionic liquid dispersive liquid-liquid microextraction-HPLC method, the former can use the USE extraction method to obtain the determination chromatogram of each compound, while the latter is a chromatogram with multiple peaks, including a variety of substances, which is not easy to distinguish. In general, the HPLC-QqLIT-MS/MS method is more suitable for the simultaneous detection of multiple compounds and has higher resolution. In the research on the determination of sulfonamides in food by LC-MS/MS, the overall effect of the chromatographic peaks obtained by the SPE extraction method is good, but the peaks of the three substances are stuck or overlapped together, which is inconvenient to observe and calculate the final result, affecting its accuracy.

In the determination of aflatoxin in food, the HPLC-FLD method and the LC-ESI-QTOF-MS/MS method also have similar flow rates, so they have little effect on the peak area, and the standard solution is also measured first. Therefore, it is easier to compare under this condition. It can be clearly seen in Figure 5 that the LC-ESI-QTOF-MS/MS method has a higher sharpness and a faster peak time, which is also due to the combination with the QTOF analyzer, which is combined use.

### 4.2. Recovery and Precision Analysis

The precision of LC-QTOF-MS was 1.0-18.1%, which was similar to that of LC-MS/MS with 3.0-19.5%, but the average recovery was 70-120%, which was higher than that of LC-MS/MS with 89-114%. It can be seen that the combination of the QTOF analyzer can also improve the recovery and precision of liquid chromatography.

In experiments for the determination of aflatoxins, the precision of the LC-MS/MS method was less than 11% and the recovery was 50-120%. The precision of the HPLC-FD method was 1.2-14.3%, and the recovery was 73-110%. The precision when analyzed by immunomagnetic solid-phase extraction coupled with UHPLC-MS/MS was less than 15.2%, and the recovery was 84.5–112.7%. By comprehensively comparing the above data, the lower the precision, the higher the average recovery, the better, so it is very desirable to use immunomagnetic solid-phase extraction on the basis of UHPLC-MS/MS.

### 4.3. Column Size and Particle Size

In terms of column selection, if the inner diameter of the column is halved, the sensitivity increases by a factor of four to five (assuming the same injection volume). For example, injecting the same amount of sample into a 2.1 mm id column produces peaks that are about 5 times higher than injection into a 4.6 mm id column. Parameters such as column efficiency, number of theoretical plates, backpressure, and analysis time are independent of the reduction in column ID as long as the linear flow rate remains constant.

In the separation process, the following sections pursue narrower peak broadening and the best column efficiency under the condition of approximate retention time. For this, we refer to the Van Deemter equation, which is the most famous chromatographic equation to date [29]. This equation expresses the change in column height equivalent to one theoretical plate (HETP) with linear mobile phase velocity:

(1) $$\begin{array}{c} H=A+\frac{B}{u}+C\times u. \end{array}$$

In the above formula, *H* is the height of the theoretical plate, which represents the peak broadening in the separation process. *u* (longitudinal molecular diffusion) is related to the inner diameter of the column and the flow rate of the mobile phase, and *C* × *u* (mass transfer resistance) is related to the particle size of the filler and the flow rate of the mobile phase. According to the calculation, we can obtain an optimal flow rate when *A*, *B*, and *C* are fixed values. For example: the optimal flow rate *u*0 of a column with a diameter of 4.6 mm and a particle size of 5 *μ*m is 1 mL/min. However, according to the data in Tables 1–3, the 4.6 mm diameter, 5 *μ*m particle size column has different flow rates. In the determination of acrylamide, the actual flow rate is 0.4 mL/min, which is less than the optimum flow rate. In the determination of sulfonamides, the actual flow rate is 0.2 mL/min, which is also less than the optimum flow rate. In the determination of aflatoxin, the actual flow rate is 1.2 mol/min, 2 mol/min, and 2-3 mol/min; these three data are larger than the optimal flow rate. So, the following sections will discuss the effect of the actual flow rate on the column efficiency (peak broadening) when the actual flow rate is greater than *u*0 and less than *u*0.

According to Figure 6 and formulas, we can conclude that when the actual flow rate is less than *u*0, *B*/*u* (longitudinal molecular diffusion) plays a major role on the plate height, *C* × *u* (mass transfer resistance) plays a secondary role on the plate height, and *A* (vortex diffusion) has a negligible effect on plate height. Therefore, under this condition, the larger the actual flow rate, the lower the theoretical plate height, and the higher the column efficiency. When the flow rate is greater than *u*0 and the actual flow rate is greater than *u*0, *C* × *u* (mass transfer resistance) plays a major role in the height of the tray, and *A* (vortex diffusion) plays a secondary role in the tray. Under this condition, as the flow rate increases, the height of the theoretical plate also increases, and the column efficiency decreases slowly. In addition, at the same flow rate, the smaller the particle size of the filler, the smaller the height of the theoretical plate, and the better the column efficiency. It can be inferred that the HPLC-FD method used in the determination of aflatoxin is superior to HPLC-MS/MS and HPLC-FLD. HPLC-MS/MS is superior to improved LC-MS/MS in the determination of acetamide content.

According to the above theory, it can also conclude that the newer methods such as fluorescence detection, UV detection, QTOF, or QuEChERS extraction combined with liquid chromatography are much better than the original liquid chromatography.

As for the selection of stationary phase and mobile phase, in the above liquid chromatography, mostly is reverse phase chromatography. In the process of determination, the nonpolar stationary phase such as C18 is mostly used, while the mobile phase is usually water or buffer. This combination of stationary and mobile phases is suitable for the separation of nonpolar and low-polar compounds. In the mobile phase, the commonly used water-soluble organic solvents are methanol, formic acid, ammonium formate, acetonitrile, isopropanol, acetone, tetrahydrofuran, and so on. These substances can regulate the retention time.

## 5. Conclusion

In this paper, by enumerating three types of food contaminants, referring to and citing different liquid chromatography methods in the literature to determine the indicators and the final results, a comparison was established in terms of chromatographic peaks, recovery, and accuracy, and the immobilization was summarized. For the principles for the selection of phase and mobile phase, with the increase of the molecular weight of the tested substance, the position of the peak in the chromatogram is correspondingly backward, and the analysis time is also correspondingly increased. When there are multiple compounds in the analyte, HRMS hybrid detectors such as QTOF analyzers can be used, which is more efficient and convenient than traditional QqQ and TOF. It should also have good clean-up techniques like PLE, USE, SPE, or QuEChERs [31]. Choosing the appropriate mobile phase ratio and flow rate of the stationary phase will help to enhance the symmetry of the chromatographic peak shape and the degree of separation and also help to improve the precision and recovery rate, so that a more efficient liquid chromatography technology can be established and used. The field of food safety testing has been more widely used.

## Figures and Tables

**Figure 1:** The working principle of HPLC.

**Figure 2:** Schematic diagram of chromatographic peak comparison.

**Figure 3:** Optimal chromatographic peaks of HPLC-UV.

**Figure 4:** (a) Chromatograms obtained by the PLE method and (b) the USE method.

**Figure 5:** Comparison of chromatographic peaks between HPLC-FLD and LC-ESI-QTOF-MS/MS.

**Figure 6:** Vandermuth equation image reference optimal flow rate determination [30].

**Table 1:** Liquid chromatography measurement conditions.

Compound	Food product	Chromatographic method	Column	Mobile phase	Flow rate	Ref.
Acrylamide (AM)	Potato chips	LC-MS/MS	Extrasyl ODS1 (200 × 30 mm, 5 *μ*m)	0.5% methanol : water 0.1% 2-propanolacetic acid	0.2 mL/min	[12]
Acrylamide (AM)	Rice, bread and coffee, etc.	Improved LC-MS/MS	C18 (250 × 2 mm, 5 *μ*m)	0.2% acetic acid 1% methanol	0.2 mL/min	[13]
Acrylamide (AM)	Dried fruit and edible seeds	QuEChERS extraction-LS-MS	Gemini RP C18 (250 × 2 mm, 5 *μ*m)	0.1% formic acid 0.1% MeOH : formic acid	0.25 mL/min	[14]
Acrylamide (AM)	Thermally processed seafood	HPLC-MS/MS	C18 (50 × 2 mm, 2.5 *μ*m)	Methanol, 0.1% formic acid Water-methanol	0.2 mL/min	[15]
Acrylamide (AM)	Chinese baked and fried foods	HPLC-UV	ODS-C18 (250 × 4.6 mm, 5 *μ*m)	ACN, water : 0.1% formic acid ACN	0.40 mL/min	[16]

**Table 2:** Liquid chromatography measurement conditions.

Compound	Food product	Chromatographic method	Column	Mobile phase	Flow rate	Ref.
STZ, SMR, SDZ, SPY, SMZ, SMT, SCP, SMA, SDM, SQX	Honey	LC-MS-MS	Zorbax Eclipse XDB-98 (50 × 4.6 mm, 1.8 *μ*m)	0.5% formic acid in water ACN	0.4 mL/min	[17]
STZ, SMZ, SPY, SGA, SMR, SMA, SDM, SDZ, SIX	Meat and/or egg-based baby foods	LC-QToF-MS	Poroshell 120 HILIC (150 × 3 mm, 2.7 *μ*m) 20 mM ammonium formate aqueous solution at pH	20 mM ammonium formate in water pH 3 : methanol in ACN 1 : 1 *v*/*v*	0.2 mL/min	[18]
SDZ, SDM, SMR, SMZ, SMT, SMA, SNM, STZ, SCP, TMP, SDX, SMPZ, SPY, SIX, SBZ, SQX, SCA, SPN	Aquatic products	Online SPE-UHPLC–MS/MS	F5 column (50 × 3.0 mm, 2.6 *μ*m)	0.1% formic acid in water 0.1% formic acid in ACN	0.45 mL/min	[19]
SMR, SMZ, SMA, SMPZ, SDZ, SPY, SDMX, S-STZ, SGA, SCA, SBZ, SNT, SIM, SMTZ, SQX, STZ, SIX, SDX	Animal muscle and liver	HPLC-QqLIT-MS/MS	CHPLC column Purosphers STAR C18 (150 × 4.6 mm, 5 *μ*m)	HPLC-grade water acidified with 10 mM of formic acid ACN with 10 mM of formic acid	0.2 mL/min	[20]
Sulfamethazine (STZ), sulfamonomethoxine (SMM), sulfadiazine (SDZ), SMZ, SMT	Milk	In situ magnetic ionic liquid dispersive liquid-liquid microextraction coupled with HPLC	C18-H column (250 × 4.6 mm, 5 *μ*m)	0.5% MSP-ACN (85 : 15, *v*/*v*)	0.2 mL/min	[21]

**Table 3:** Liquid chromatography measurement conditions.

Compound	Food product	Chromatographic method	Column	Mobile phase	Flow rate	Ref.
AFB1, AFB2, AFG1, AFG2	Maize	LC-MS-MS	Purospher Star RP-18 (50 × 2.1 mm, 2 *μ*m)	0.1% acetic acid-methanol (60 : 40)	0.25 mL/min	[23]
AFB1, AFB2, AFG1, AFG2	Wheat, soybeans, peanuts, etc.	LC -ESI-QTOF-MS/MS	ZORBAX Eclipse XBD-C18 (100 × 2.1 mm, 1.8 *μ*m)	1% formic acid and 2 mM ammonium formate in water 1% formic acid in methanol	0.3 mL/min	[24]
AFB1, AFB2, AFG1, AFG2	Glycyrrhiza uralensis	HPLC-MS/MS	C18-H column (250 × 4.6 mm, 5 *μ*m)	0.5% MSP-ACN (85 : 15, *v*/*v*)	2 mL/min	[25]
AFM2, AFM1, AFB2, AFB1	Milk	Micro-SPE-HPLC-UV	C18 Hypersil gold (250 × 4.6 mm, 5 *μ*m)	Acetonitrile : methanol 3 : 2 (*v*/*v*)	1.2 mL/min	[26]
AFB1, AFB2, AFG1, AFG2	Pistachios and groundnuts	HPLC-FLD	ACE 5 C18, 100 A (250 × 4.6 mm, 5 *μ*m)	Water-acetonitrile-ethanol (6/2/3, *v*/*v*/*v*)	2-3 mL/min	[27]

## Data Availability

The datasets used and/or analyzed during the current study are available from the corresponding author on reasonable request.
